# A Flexible Bayesian Parametric Proportional Hazard Model: Simulation and Applications to Right-Censored Healthcare Data

**DOI:** 10.1155/2022/2051642

**Published:** 2022-06-02

**Authors:** Abdisalam Hassan Muse, Oscar Ngesa, Samuel Mwalili, Huda M. Alshanbari, Abdal-Aziz H. El-Bagoury

**Affiliations:** ^1^Department of Mathematics (Statistics Option), Pan African University Institute for Basic Science Technology and Innovation (PAUSTI), Nairobi 62000 00200, Kenya; ^2^Department of Mathematics and Physical Sciences, Taita Taveta University, Voi 635-80300, Kenya; ^3^Department of Statistics and Actuarial Sciences, Jomo Kenyatta University of Agriculture and Technology (JKUAT), Nairobi, Kenya; ^4^Department of Mathematical Sciences, College of Science, Princess Nourah bint Abdulrahman University, P.O. Box 84428, Riyadh 11671, Saudi Arabia; ^5^Basic Science Department, Higher Institute of Engineering and Technology, El-Mahala El-Kubra, Egypt

## Abstract

Survival analysis is a collection of statistical techniques which examine the time it takes for an event to occur, and it is one of the most important fields in biomedical sciences and other variety of scientific disciplines. Furthermore, the computational rapid advancements in recent decades have advocated the application of Bayesian techniques in this field, giving a powerful and flexible alternative to the classical inference. The aim of this study is to consider the Bayesian inference for the generalized log-logistic proportional hazard model with applications to right-censored healthcare data sets. We assume an independent gamma prior for the baseline hazard parameters and a normal prior is placed on the regression coefficients. We then obtain the exact form of the joint posterior distribution of the regression coefficients and distributional parameters. The Bayesian estimates of the parameters of the proposed model are obtained using the Markov chain Monte Carlo (McMC) simulation technique. All computations are performed in Bayesian analysis using Gibbs sampling (BUGS) syntax that can be run with Just Another Gibbs Sampling (JAGS) from the R software. A detailed simulation study was used to assess the performance of the proposed parametric proportional hazard model. Two real-survival data problems in the healthcare are analyzed for illustration of the proposed model and for model comparison. Furthermore, the convergence diagnostic tests are presented and analyzed. Finally, our research found that the proposed parametric proportional hazard model performs well and could be beneficial in analyzing various types of survival data.

## 1. Introduction

The healthcare domain has evolved significantly in recent years as a result of computational developments. The use of Bayesian statistics in healthcare has encouraged the application of computational developments, providing a powerful and versatile alternative to traditional methodologies used in healthcare [1]. The progress of Bayesian approaches in healthcare aims to make an individual's life more affordable and comfortable, similar to how smartphones have made life easier [2]. Despite the fact that the idea of applying computational Bayesian statistics to survival analysis dates back to the 19th century, McMC techniques are now garnering more attention in the literature because of abundant and cheap computation [3]. The application of deep learning to the context of parametric survival models was discussed by [4]. Through an efficient training process, the quality of the developed system improves. Data portioning is done three times to confirm the trained algorithms (training-testing-validation) [5]. The main goal of this article is to present the Bayesian parametric proportional hazard model using BUGs syntax.

The statistical analysis of survival data is an essential topic in many fields, including medicine, biology, environmental science, healthcare, economics, engineering, social science, and epidemiology, among others. Probability distributions serve as the foundation for survival models. The family of distributions can be parametric, semiparametric, or nonparametric. The parametric survival models lead to more efficient and smaller standard errors of the estimates than semiparametric and nonparametric models [6] if the distributional assumption is correct, to be more specific.

In analyzing survival data, parametric survival models are crucial. The benefits of using parametric survival models include the following: (1) handling all types of censored data (left, right, interval, double, and middle); (2) application of survival analysis in a healthcare care problem and (3) producing better estimation when you have a theoretical expectation of the baseline hazard; also, (4) they can apply random effects—frailty models—and can also be used to estimate expected lives, not only hazard ratios like the accelerated failure time models [7].

The proportional hazards (PH) model, in which covariates affect the hazard rate function, and the accelerated failure time (AFT) model, in which covariates affect both the hazard rate and time scale, are the two most common methods for developing parametric regression models for survival data [8]. However, other class of models have also been proposed such as the accelerated hazard (AH) model [9] and the proportional odds (PO) model [10].

One of the first steps in using a parametric approach to model survival data is to choose a suitable baseline distribution that can capture significant features of the observations of interest. Certain probability distributions are widely used in the modelling of survival data. Only a few are closed under the proportional hazard model, and none are flexible enough to describe a wide range of survival data [11]. Most of the distributions closed under the PH assumption fails to model a nonmonotone (i.e., bathtub and unimodal) survival data sets.

The log-logistic (LL) distribution has a wide range of applications in survival data analysis and can accommodate unimodal survival data sets. The distribution is closed under both proportionality odds (PO) and multiplication of failure time (AFT) frameworks [7]. It is not a PH model, but an AFT model. However, when the log-logistic distribution is generalized, it has the appealing feature of being a member of all classes of parametric hazard-based regression models of the survival analysis because its failure rate function is quite versatile and its cumulative hazard function (chf) has a tractable form.

Extensive efforts have been made over the last decades to extend classical distributions to use as a baseline distribution for parametric hazard-based regression models. Many modifications to the LL distribution have been introduced to make it more adaptable to a wide range of hazard shapes [12–16]. The generalized log-logistic distribution (GLL) is one such model, which modifies the log-logistic distribution by inducing an additional shape parameter [17]. The model is tractable and closed under the PH assumption and can account for both nonmonotone and monotone hazard rates [11]. On the other hand, recent computational advances have advocated for the use of Bayesian techniques in the field of survival and reliability analysis.

The motivating ideas behind our work on Bayesian parametric proportional hazard (PH) model with GLL baseline hazard are as follows: (i) despite the fact that there are some classical distributions closed under the PH framework, none of which is flexible enough to incorporate both monotone and nonmonotone hazard rate; (ii) Bayesian inference does not rely on asymptotic approximation for statistical inference; (iii) the availability of software makes Bayesian implementation for hazard-based complicated models relatively more straightforward and simple than classical inference [18]; (iv) parametric PH model may lead to more precise estimates than the semiparametric PH model; and, last but not the least, (v) the use of generalized distributions that can capture both monotone and nonmonotone hazard rate functions is what makes our work unique and more appealing to biostatisticians, epidemiologists, healthcare workers, and other applied researchers in multiple disciplines.

To the best of author's knowledge, no Bayesian inferences study has been conducted on the PH model with generalized log-logistic baseline hazard. As a result, in this paper, we consider the Bayesian inference for the generalized log-logistic proportional hazard model, beginning with the PH model formulation and assumptions, revising the generalized log-logistic distribution, and verifying that the GLL distribution is closed under the PH framework. In addition, we discuss the inferential procedures and how to obtain the classical and Bayesian estimators for the model's parameters. We also compare the proposed model to other existing distributions closed under the PH framework, and one interesting feature of this model is that it can incorporate different hazard rate shapes. Hence, the formulation of the parametric PH model and its lifetime function, the inferential procedures using both classical and Bayesian approaches, and the development of the computational algorithms to fit the proposed PH model and its competing models using RJAGS in R software are the novelty of this study.

The article is structured as follows: the PH model formulation, assumptions, and its probabilistic functions are discussed in Section 2.  Section 3 revises the most common probability distributions closed under the PH model.  Section 4 presents the proposed baseline hazard function which is a generalized log-logistic (GLL) distribution. The GLL distribution under the PH model is presented in Section 5.  Section 6 discusses the inferential procedures of the proposed model. In Section 7, we present an McMC simulation study to assess the performance of the proposed model.  Section 8 presents the application of the proposed model to two right-censored cancer data sets with monotone and nonmontone hazard rates. In addition, the convergence diagnostics of the McMC techniques were discussed. The Bayesian model selection criterion is presented in Section 9. Finally, in the final portion, the article's concluding notes are offered, and some future works are mentioned.

## 2. PH Model Formulation and Assumptions

In many real-life applications, survival times are affected by explanatory variables. The explanatory variable vector is related to response variable through a regression model. An important aspect of survival modelling is the inclusion of explanatory variables. The hazard-based regression models can be formulated in a number of ways. One of the most frequently used method is the proportional hazard (PH) model formulation.

PH models play an essential role in analyzing time-to-event data and are broadly used in survival and reliability analysis as well as in joint modelling of survival and longitudinal data [7]. It is the most popular parametric model in medical studies and clinical trials because of the existence of a semiparametric PH hazard model which is robust against the distributional assumption of the survival time. The parametric PH model is given with the similar form to the Cox PH model. It is the parametric form of the Cox PH models [6].

### 2.1. PH Model Formulation

The parametric proportional hazard (PH) models are formulated using a defined baseline hazard and a link function *ψ*(**x** ′*β*) for the covariates which is defined as follows:

(1) $$\begin{array}{c} \psi \left(x{\;}^{\prime }\beta \right)>0,\;\forall x\neq 0,\\ \psi \left(x{\;}^{\prime }\beta \right)\text{is a monotone function that has a one}‐\text{to-one correspondence,}\\ \psi \left(0\right)=1. \end{array}$$

The most commonly found option for the link function *ψ*(**x** ′*β*) is the exponential exp(**x**^**'**^*β*)  (or log-linear) function. In this work, we define the PH model with the assumption that *ψ*(**x** ′*β*)=exp(**x** ′*β*). 

### 2.2. PH Assumptions

The PH model assumption is that the effect of covariates is to increase or decrease the hazard rate function by a proportionate amount which does not depend on *t*. The assumption of the PH model can be defined as follows:

(2) $$\begin{array}{c} h\left(t;x\right)=\;h_{0}\left(t\right)\psi \left(x{\;}^{\prime }\beta \right)=h_{0}\left(t\right)\exp\left(x{\;}^{\prime }\beta \right)\;=h_{0}\left(t\right)e^{x^{\prime }\beta }, \end{array}$$

where *h*_0_(*t*) is called the baseline hazard.

Simplifying, we get,

(3) $$\begin{array}{c} h\left(t|x\right)=\;h_{0}\left(t\right)\text{exp}\left(\beta_{1}x_{1}+\beta_{2}x_{2}+\ldots +\beta_{p}x_{p}\right). \end{array}$$

The main difference between the Cox PH model and the parametric PH model is that the baseline hazard function is assumed to follow a specific distribution when it is fitted to the data. Using equation (2), we can see that the hazard ratio (HR) comparing any two specifications of the covariates, for example, (**x** and **x**^**∗**^) is

(4) $$\begin{array}{c} HR\left(x,\mathrm{x*},h_{0},\beta \right)=\frac{h\left(t|x,\;\beta \right)}{h\left(t|x^{*},\;\beta \right)}=\;\frac{h_{0}\left(t|x\right)\text{exp}\left(\mathrm{\beta x}{\;}^{\prime }\right)}{h_{0}\left(t|x\right)\text{exp}\left(\beta x^{{*}^{'}}\right)}=\;\exp\left[{\left(x{\;}^{\prime }-\;x^{{*}^{'}}\right)}^{T}\beta \right]. \end{array}$$

The above equation shows us that the baseline hazards cancel each other from this ratio, so the hazard rate for one individual is proportional to the hazard rate for any other individual. On the other hand, the proportionality constant is independent of time which makes the main assumption of this model [6]. As a result, the model is known as the proportional hazard (PH) model in the literature.

Unlike most parametric regression models including accelerated failure time (AFT) models, PH models does not include an intercept [19]. More properly, the vector **X** in the PH model is not assumed to have *x* ≡ 1. An intercept would get confounded with the baseline hazard function *h*_0_.

### 2.3. Lifetime Functions Describing the PH Model

The five frequent representatives of a lifetime distribution function that are used to characterize the PH model are addressed in this section.

#### 2.3.1. Hazard Rate Function of the PH Model

In the PH analysis, one of the most important lifetime functions is the concept of the hazard rate function (hrf). The hazard rate function *h*(*t|x*), abbreviated by hrf, also called the instantaneous failure rate or as force of mortality of a PH model is of the form:

(5) $$\begin{array}{c} h\left(t;x\right)=\;h_{0}\left(t\right)\psi \left(x{\;}^{\prime }\beta \right)=h_{0}\left(t\right)\exp\left(x{\;}^{\prime }\beta \right)\;=h_{0}\left(t\right)e^{x^{\prime }\beta }. \end{array}$$

#### 2.3.2. Cumulative Hazard Function of the PH Model

The hazard or survival functions, rather than the cumulative distribution or probability density function, are typically used in the PH analysis of survival data. The hazard rate function is used to interpret the most common survival regression models; however, the cumulative hazard function (chf), also known as the integrated hazard rate function, can be easily written down. Hence, the chf of a PH model takes the following form:

(6) $$\begin{array}{c} H\left(t|x\right)=\;\overset{t}{\underset{0}{\int }}h\left(s;x\right)\text{ds }=\;e^{x^{\prime }\beta }\;\overset{t}{\underset{0}{\int }}h_{0}\left(s\right)\text{ ds }=\;e^{x^{\prime }\beta }\;H_{0}\left(t\right).\; \end{array}$$

#### 2.3.3. Survival Function of the PH Model

The survivor function (sf) for a PH model can be derived using the following relationship between survival function and the hazard rate function. Hazard function is given by

(7) $$\begin{array}{c} h\left(t|x\right)=\frac{f\left(t|x\right)}{S\left(t|x\right)}. \end{array}$$

Cumulative hazard function:

(8) $$\begin{array}{c} H\left(t|x\right)=\overset{t}{\underset{0}{\int }}h\left(u\right)\text{du}=\;\overset{t}{\underset{0}{\int }}\frac{f\left(u\right)}{S\left(u\right)}\text{du}=\overset{t}{\underset{0}{\int }}\frac{-\text{dS}\left(u\right)}{S\left(u\right)}\text{du}=\;-\text{log}\left\{S\left(t\right)\right\},\\ f\left(t|x\right)=h\left(t|x\right)S\left(t|x\right)=h\left(t|x\right)\exp\left\{-H\left(t|x\right)\right\}. \end{array}$$

Using the above expressions, we can easily find

(9) $$\begin{array}{c} \;S\left(t|x\right)=\exp\left\{-H\left(t|x\right)\right\},\\ S\left(t|x\right)=\exp\left\{-H\left(t|x\right)\right\}=\text{exp}\left\{-\int_{0}^{t}\psi \left(x\right)h_{0}\left(t\right)\;dt\right\},\\ =\text{ exp}\left\{-\psi \left(x\right)\int_{0}^{t}h_{0}\left(t\right)\;dt\right\},\;\\ ={\left[\text{exp}\left\{-\int_{0}^{t}h_{0}\left(t\right)\;dt\right\}\;\right]}^{\psi \left(x\right)}\;,\;\\ ={\left[\;S_{0}\left(t\right)\right]}^{\psi \left(x\right)}. \end{array}$$

#### 2.3.4. Cumulative Distribution Function of the PH Model

The cdf of the PH model, also known as the lifetime distribution function, is given by

(10) $$\begin{array}{c} F\left(t\right)=1-S\left(t\right)=1-\;\exp\left\{-H\left(t\right)\right\},\\ F\left(t\right)=1-\;{\left[S_{0}\left(t\right)\right]}^{\psi \left(x\right)}. \end{array}$$

#### 2.3.5. Probability Density Function of the PH Model

The pdf or the failure density function of the PH model is defined as

(11) $$\begin{array}{c} f\left(t\right)=f_{0}\left(t\right)\psi \left(x\right){\left[\;S_{0}\left(t\right)\right]}^{\psi \left(x\right)-1}. \end{array}$$

The five representatives used here were chosen for their special meaning for lifetime data, their intuitive appeal, their utility in survival data analysis, and, last but not the least, their popularity in probability theory and statistics.

The PH model can be formulated without assuming a probability distribution for survival times, and this leads to the well-known Cox PH model [20]. On the other hand, assuming a probability distribution for survival times leads to the fully parametric PH model. The most common parametric survival models used are as follows: exponential, Weibull, Gompertz, log-logistic, log-normal, gamma, and the generalized gamma distributions. Only the exponential, Weibull, and Gompertz distributions are used for the PH model. The log-logistic and the log-normal distributions are not closed under the PH framework. Weibull distribution is the only one that is closed under both parametric AFT and PH models.

## 3. Distributions Closed under PH Framework

In this section, we present most common parametric distributions that are closed under the PH framework and are used to analyze survival data. These distributions have been studied and used in various contexts in the literature.

### 3.1. Exponential PH Model

Exponential distribution is a continuous probability distribution with only one unknown parameter *k*. It is the simplest distribution for lifetime distribution models. The distribution is not flexible enough to describe commonly encountered hazard rate shapes for survival data. The pdf, cdf, sf, hrf, and chf of the exponential random variable are, respectively, as follows.

Let *X* ~ exponential(*k*),

(12) $$\begin{array}{c} f\left(t\right)=\;k\;\exp\left\{-\text{kt}\right\},\\ F\left(t\right)=\;1-\exp\left\{-\text{kt}\right\},\\ S\left(t\right)=\;\exp\left\{-\text{kt}\right\},\\ h\left(t\right)=\;k,\\ H\left(t\right)=-\text{log}S\left(t\right)=\;-\text{log}\left(\exp\left\{-\text{kt}\right\}\right.=kt, \end{array}$$

where *k* > 0 is the scale parameter and *t* ≥ 0. A short value of *k* shows low risk and long survival, where a large value shows high risk and short survival. For the PH model, the exponential baseline hazard is

(13) $$\begin{array}{c} h\left(t\right)=\;k. \end{array}$$

So, according to the formulation of the PH framework, the hazard rate for an individual with covariate vector *x* and link function *ψ*(*x*) is

(14) $$\begin{array}{c} h\left(t\right)=h_{0}\left(t\right)\;\psi \left(x\right)=k.\psi \left(x\right)\;. \end{array}$$

Applying the log-linear function *ψ*(**x** ′*β*)=exp(**x** ′*β*) , we can simplify into

(15) $$\begin{array}{c} h_{EPH}\left(t\right)=k.\;\exp\left(x^{'}\beta \right)\;=k.\;\exp\left(\beta_{1}x_{1}+\beta_{2}x_{2}+\ldots +\beta_{p}x_{p}\right). \end{array}$$

In this equation, the hrf has the exponential distribution with scale parameter k.  exp(**x** ′*β*) which indicates that the PH assumption is satisfied with the exponential distribution. It is worth mentioning that the exponential distribution is often found to be inadequate to describe survival data. This makes the applicability of this distribution fairly limited.

The other lifetime distributions of the exponential PH model are as follows.

The survival function of the exponential PH model is

(16) $$\begin{array}{c} S_{\text{EPH}}\left(t\right)=\left[\exp\left\{-kt\right\}\right]{\;}^{\exp\left(x{\;}^{\prime }\beta \right)\;}. \end{array}$$

The pdf of the exponential PH model is

(17) $$\begin{array}{c} f_{\text{EPH}}\left(t\right)=\;k\;\exp\left\{-kt\right\}\exp\left(x{\;}^{\prime }\beta \right)\left[\exp\left\{-kt\right\}\right]{\;}^{\exp\left(x{\;}^{\prime }\beta \right)-1}. \end{array}$$

The cdf of the exponential PH model is

(18) $$\begin{array}{c} F_{\text{EPH}}\left(t\right)=1-\;\left[\exp\left\{-kt\right\}\right]{\;}^{\exp\left(x^{'}\beta \right)}. \end{array}$$

The chf of the exponential PH model is

(19) $$\begin{array}{c} H_{\text{EPH}}\left(t\right)=kt\;\exp\left(x{\;}^{\prime }\beta \right). \end{array}$$

### 3.2. Gompertz PH Model

Gompertz distribution is named after Benjamin Gompertz, a British mathematician and actuary, who developed it in 1825. It is a continuous probability distribution used for modelling adult life spans and other application under different disciplines such as actuarial science, demography, survival, and reliability analysis. This distribution is flexible and can be skewed both in right and in left. The pdf, cdf, sf, hrf, and chf of the exponential random variable are, respectively, as follows.

Let *X* ~ Gompertz(*k*,  *α*),

(20) $$\begin{array}{c} f\left(t\right)=\;\alpha k.e^{tk}\exp\left\{-\;\alpha \left(e^{tk}-1\right.\right\},\;t\in \left[0,\infty \right),\\ F\left(t\right)=\;1-\exp\left\{-\;\alpha \left(e^{tk}-1\right.\right\},\\ S\left(t\right)=\;\exp\left\{-\;\alpha \left(e^{tk}-1\right.\right\},\\ h\left(t\right)=\;=\;{\;\alpha \text{ke}}^{tk},\\ H\left(t\right)=-\text{log}S\left(t\right)=\;-\log\left[\exp\left\{-\;\alpha \left(e^{tk}-1\right.\right\}\right]=\;\alpha \left(e^{tk}-1\right), \end{array}$$

where *k* > 0 is the rate parameter, *α* > 0  is the shape parameter,  and *t* ≥ 0. When *k* ≥ 0, the survival time then has an exponential distribution; therefore, Gompertz distribution is a generalization of exponential distribution. For the PH model, the Gompertz baseline hazard rate function is given by

(21) $$\begin{array}{c} h\left(t\right)={\alpha \text{ke}}^{tk}. \end{array}$$

So, according to the formulation of the PH framework, the hazard rate for an individual with covariate vector *x* and link function *ψ*(*x*) is

(22) $$\begin{array}{c} h\left(t\right)=h_{0}\left(t\right)\;\psi \left(x\right)=\;\alpha \text{k}.e^{tk}.\psi \left(x\right). \end{array}$$

Applying the log-linear function *ψ*(**x** ′*β*)=exp(**x** ′*β*) , we can simplify into

(23) $$\begin{array}{c} h_{\text{GoPH}}\left(t\right)=\;\alpha k.e^{tk}.\;\exp\left(x{\;}^{\prime }\beta \right)\;=\;\alpha k.e^{tk}.\;\exp\left(\beta_{1}x_{1}+\beta_{2}x_{2}+\ldots +\beta_{p}x_{p}\right). \end{array}$$

In the above equation, it is straightforward that the PH property is satisfied. However, the Gompertz PH model is rarely used in the real-life applications.

The other lifetime distributions of the Gompertz PH model are as follows: the survival function of the Gompertz PH model is

(24) $$\begin{array}{c} S_{\text{GoPH}}\left(t\right)=\left[\exp\left\{-\;\alpha \left(e^{tk}-1\right.\right\}\right]{\;}^{\exp\left(x{\;}^{\prime }\beta \right)\;}. \end{array}$$

The pdf of the Gompertz PH model is

(25) $$\begin{array}{c} f_{\text{GoPH}}\left(t\right)=\;\alpha k.e^{tk}\exp\left\{-\;\alpha \left(e^{tk}-1\right.\right\}\exp\left(x{\;}^{\prime }\beta \right)\left[\exp\left\{-\;\alpha \left(e^{tk}-1\right.\right\}\right]{\;}^{\exp\left(x{\;}^{\prime }\beta \right)-1}. \end{array}$$

The cdf of the Gompertz PH model is

(26) $$\begin{array}{c} F_{\text{GoPH}}\left(t\right)=\;1-\;\left[\exp\left\{-\;\alpha \left(e^{tk}-1\right.\right\}\right]{\;}^{\exp\left(x{\;}^{\prime }\beta \right)\;}. \end{array}$$

The chf of the Gompertz PH model is

(27) $$\begin{array}{c} H_{\text{GoPH}}\left(t\right)=\exp\left(x{\;}^{\prime }\beta \right)\;\alpha \left(e^{tk}-1\right). \end{array}$$

### 3.3. Weibull PH Model

Weibull distribution is a generalization of the exponential distribution. It is a versatile distribution that can take on the characteristics of other types of continuous distributions. It has an additional parameter compared to the exponential. The additional parameter describes the shape of the hazard functions, based on the value of the shape parameter [21]. The pdf, cdf, sf, hrf, and chf of the Weibull random variable are, respectively, as follows.

Let *X* ~ Weibull(*k*,  *α*),

(28) $$\begin{array}{c} f\left(t\right)=\;\alpha k{\left(kt\right)}^{\;\alpha -1}\exp\left\{-{\left(kt\right)}^{\;\alpha }\right\},\\ F\left(t\right)=\;1-\exp\left\{-{\left(kt\right)}^{\;\alpha }\right\},\\ S\left(t\right)=\;\exp\left\{-{\left(kt\right)}^{\;\alpha }\right\},\\ h\left(t\right)=\;\alpha k{\left(kt\right)}^{\;\alpha -1},\\ H\left(t\right)=-\text{log}S\left(t\right)=\;-\text{log}\left(\exp\left\{-{\left(kt\right)}^{\;\alpha }\right\}\right.={\left(kt\right)}^{\alpha }, \end{array}$$

where *α* > 0 is the shape parameter and *k* > 0 is the rate parameter. The hazard rate function increases when  *α* > 1, decreases for  *α* < 1, and constant for  *α*=1. When  *α*=1, the Weibull distribution reduces to exponential. It is worth mentioning that the Weibull distribution does not accommodate nonmonotone (i.e., unimodal or bathtub) hazard rates.

For the PH model the Weibull baseline hazard is

(29) $$\begin{array}{c} h\left(t\right)=\;\alpha k{\left(kt\right)}^{\;\alpha -1}. \end{array}$$

So, according to the formulation of the PH framework, the hazard rate for an individual with covariate vector *x* and link function *ψ*(*x*) is

(30) $$\begin{array}{c} h\left(t\right)=h_{0}\left(t\right)\;\psi \left(x\right)=\;\alpha k{\left(kt\right)}^{\;\alpha -1}\psi \left(x\right)\;. \end{array}$$

Applying the log-linear function *ψ*(**x**^**'**^*β*)=exp(**x**^**'**^*β*) , we can simplify into

(31) $$\begin{array}{c} h_{\text{WPH}}\left(t\right)=\;\alpha k{\left(kt\right)}^{\;\alpha -1}\exp\left(x{\;}^{\prime }\beta \right)=\;\alpha k{\left(kt\right)}^{\;\alpha -1}\exp\left(\beta_{1}x_{1}+\beta_{2}x_{2}+\ldots +\beta_{p}x_{p}\right). \end{array}$$

In this equation, the model has the Weibull distribution with rate parameter k.  exp(**x**^**'**^*β*)  and shape parameter  *α* which indicates that the PH assumption is satisfied with the Weibull distribution with constant  *α*.

The other lifetime distributions of the PH Weibull model are as follows: the survival function of the Weibull PH model is

(32) $$\begin{array}{c} S_{\text{WPH}}\left(t\right)=\left[\exp\left\{-{\left(kt\right)}^{\;\alpha }\right\}\right]{\;}^{\exp\left(x{\;}^{\prime }\beta \right)\;}. \end{array}$$

The pdf of the Weibull PH model is

(33) $$\begin{array}{c} f_{WPH}\left(t\right)=\;\alpha k{\left(kt\right)}^{\;\alpha -1}\exp\left\{-{\left(kt\right)}^{\;\alpha }\right\}\exp\left(x{\;}^{\prime }\beta \right)\left[\exp\left\{-{\left(kt\right)}^{\;\alpha }\right\}\right]{\;}^{\exp\left(x^{'}\beta \right)-1\;}.\; \end{array}$$

The cdf of the Weibull PH model is

(34) $$\begin{array}{c} F_{\text{WPH}}\left(t\right)=1-\;\left[\exp\left\{-{\left(kt\right)}^{\;\alpha }\right\}\right]{\;}^{\exp\left(x{\;}^{\prime }\beta \right)}\;. \end{array}$$

The chf of the Weibull PH model is

(35) $$\begin{array}{c} H_{\text{WPH}}\left(t\right)=\exp\left(x{\;}^{\prime }\beta \right){\left(kt\right)}^{\;\alpha }. \end{array}$$

## 4. Parametric Baseline Hazard

The parametric baseline hazard function is essential because it determines which hazard shapes can be captured by the proportional hazard (PH) model. Most classical distributions that are closed under the PH framework, such as the exponential, Weibull, and Gompertz distributions, are incapable of accommodating unimodal hazard shapes. As a result, it is worth looking into some modifications to the classical distributions that can account for both monotone and nonmonotone hazard rates.

In this paper, we consider the Bayesian inference for the parametric PH models with generalized log-logistic (GLL) baseline. The GLL is a flexible survival distribution proposed by [11]. This distribution has a characteristic similar to those of the log-logistic distribution. Also, the advantage of the GLL distribution is that it approaches to Weibull in the limit. These properties allowed the GLL to handle both monotone and nonmonotone hazard functions, and also it makes to be a baseline distribution that is closed under both AFT and PH model [22] like the Weibull distribution. The distribution is adaptable, and the two shape parameters enable a wide range of hazard shapes. It also includes a variety of important distributions such as the exponential, Weibull, Burr XII, and log-logistic distributions. In addition, when compared to competitors, it is relatively tractable. We refer to, for more information on the distribution and its properties, [17].

For a positive-valued random variable *T*, the hrf of the GLL distribution with three unknown parameters *k* > 0,  *α* > 0, *η* > 0  is given by

(36) $$\begin{array}{c} h\left(t;\;\theta \right)=\;\frac{\alpha k{\left(kt\right)}^{\alpha -1}}{\left[1+{\left(\eta t\right)}^{\alpha }\right]}=\frac{\alpha k^{\alpha }t^{\alpha -1}}{\left[1+{\left(\eta t\right)}^{\alpha }\right]}\;,\;t\geq 0,\;k,\;\alpha ,\;\eta >0\;. \end{array}$$

The chf of the GLL distribution is given by

(37) $$\begin{array}{c} H\left(t;\;\theta \right)=\;\frac{k^{\alpha }}{\eta^{\alpha }}\text{ log }\left[1+{\left(\eta t\right)}^{\alpha }\right],\;t\geq 0,\;k,\;\alpha ,\;\eta >0. \end{array}$$

The distribution function of the GLL model is of the form:

(38) $$\begin{array}{c} F\left(t;\;\theta \right)=1-{\left[1+{\left(\eta t\right)}^{\alpha }\right]}^{-\;k^{\alpha }/\eta^{\alpha }}\;,\;t\geq 0,\;k,\;\alpha ,\;\eta >0. \end{array}$$

The survival function (sf) of the GLL model is given by

(39) $$\begin{array}{c} S\left(t;\;\theta \right)=\;{\left[1+{\left(\eta t\right)}^{\alpha }\right]}^{-\;k^{\alpha }/\eta^{\alpha }}\;,\;t\geq 0,\;k,\;\alpha ,\;\eta >0\;, \end{array}$$

where *k* > 0,  *α* > 0,  and *η* > 0  are parameters and *θ*=(*k*,  *α*,  *η*)′.

The quantile function of the GLL model is given by

(40) $$\begin{array}{c} X_{q=\;}F^{-1}\left(q;\;k,\alpha ,\;\eta \right)=\frac{{\left\{{\left[1/1-q-1\right]}^{\eta^{\alpha }/k^{\alpha }}-1\right\}}^{1/\alpha }}{\eta }\;,\;0\leq q<1. \end{array}$$

The reverse cumulative hazard rate function is expressed as follows:

(41) $$\begin{array}{c} H_{0}^{-1}\left(u;\;\theta \right)=\frac{{\left(e^{\eta^{\alpha }k^{-\alpha }u}-1\right)}^{1/\alpha }}{\eta }. \end{array}$$

Figure 1 illustrates shapes that the failure rate function can accept such as constant, increasing, decreasing, V-shape, and unimodal among others.

## 5. The Proposed PH Model

For the PH model, the generalized log-logistic baseline hazard is

(42) $$\begin{array}{c} h\left(t\right)=\;\frac{\alpha k{\left(kt\right)}^{\alpha -1}}{\left[1+{\left(\eta t\right)}^{\alpha }\right]}\;. \end{array}$$

So, according to (2), the hazard rate for an individual with covariate vector *x* and link function *ψ*(*x*) is

(43) $$\begin{array}{c} h\left(t\right)=h_{0}\left(t\right)\;\psi \left(x\right)=\frac{\alpha k{\left(kt\right)}^{\alpha -1}}{\left[1+{\left(\eta t\right)}^{\alpha }\right]}\;\psi \left(x\right)\;.\; \end{array}$$

Applying the log-linear function *ψ*(**x** ′*β*)=exp(**x** ′*β*), we can simplify into

(44) $$\begin{array}{c} h_{\text{GLLPH}}\left(t\right)=\frac{\alpha k{\left(kt\right)}^{\alpha -1}}{\left[1+{\left(\eta t\right)}^{\alpha }\right]}\;\exp\left(x{\;}^{\prime }\beta \right)\;=\frac{\alpha k^{\alpha }t^{\alpha -1}}{\left[1+{\left(\eta t\right)}^{\alpha }\right]}\;\exp\left(x{\;}^{\prime }\beta \right)\;=\;\frac{\alpha {\left(k.\;\exp\;{\left(x{\;}^{\prime }\beta \right)}^{1/\alpha }\right)}^{\alpha }t^{\alpha -1}}{\left[1+{\left(\eta t\right)}^{\alpha }\right]}=\;\frac{\alpha k^{*}{\;}^{\alpha }t^{\alpha -1}}{\left[1+{\left(\eta t\right)}^{\alpha }\right]}. \end{array}$$

In this equation, the hrf can be recognized as a generalized log-logistic distribution as well, but contrary to (36), the rate parameter is *k*^*∗*^=*k*.  exp  (**x** ′*β*)^1/*α*^  and shape parameters are *α* and *η* which indicates that the PH assumption is satisfied with the GLL distribution and the proposed model is closed under the PH framework.

The other lifetime distribution functions for the GLL PH model are as follows: the survivor function of the GLL PH model is

(45) $$\begin{array}{c} S_{\text{GLLPH}}\left(t\right)=\left[{\left[1+{\left(\eta t\right)}^{\alpha }\right]}^{-k^{\alpha }/\eta^{\alpha }}\right]{\;}^{\exp\left(x{\;}^{\prime }\beta \right)\;}. \end{array}$$

The pdf of the GLL PH model is

(46) $$\begin{array}{c} f_{\text{GLLPH}}\left(t\right)=\frac{\beta c{\left(ct\right)}^{\beta -1}}{{\left[1+{\left(\eta t\right)}^{\beta }\right]}^{c^{\beta }/\eta^{\beta }+1}}\exp\left(x{\;}^{\prime }\beta \right){\left[{\left[1+{\left(\eta t\right)}^{\alpha }\right]}^{k^{\alpha }/\eta^{\alpha }}\right]}^{\exp\left(x{\;}^{\prime }\beta \right)\;-1}. \end{array}$$

The cdf of the GLL PH model is

(47) $$\begin{array}{c} F_{\text{GLLPH}}\left(t\right)=1-\;\left[{\left[1+{\left(\eta t\right)}^{\alpha }\right]}^{-k^{\alpha }/\eta^{\alpha }\;}\right]{\;}^{\exp\left(x{\;}^{\prime }\beta \right)}. \end{array}$$

The chf of the GLL PH model is

(48) $$\begin{array}{c} H_{\text{GLLPH}}\left(t\right)=\exp\left(x{\;}^{\prime }\beta \right)\frac{k^{\alpha }}{\eta^{\alpha }}\;log\;\left[1+{\left(\eta t\right)}^{\alpha }\right]. \end{array}$$

## 6. Model Inference

We discuss the classical approach (using maximum likelihood (MLE)) and Bayesian approach (assuming noninformative priors) estimation techniques for the proposed parametric PH model parameters in this section.

### 6.1. MLE for Right Censored Survival Data

We examine the challenge of estimating the proposed model's distributional parameters and regression coefficients for right-censored survival data in this section. Because of its appealing qualities, such as consistency, asymptotic efficiency, asymptotic unbiasedness, and asymptotic normality, MLE is one of the most common strategies for estimating the parameters of hazard-based regression models. Let there be *n* individuals with lifetimes represented by *T*_1_, *T*_2_,   …,  *T*_*n*_.  Assuming that the data are subject to right censoring, we observe *t*_*i*_=min(*T*_*i*_, *C*_*i*_), where *C*_*i*_ > 0 corresponds to a potential censoring time for individual *i*. Allow *δ*_*i*_=I(*T*_*i*_, *C*_*i*_) that equals 1 if  *T*_*i*_ ≤ *C*_*i*_ and 0 otherwise.

Suppose that a right-censored random sample with data *D*=(*t*_*i*_,  *δ*_*i*_,  **x**_**i**_), *i*=1,2,…, *n*, is available, where *t*_*i*_ is the censoring time or a survival time according to whether *δ*_*i*_=0 or 1, respectively, and **x**_**i**_=*x*_1_, *x*_2_,   …,  *x*_*n*_  is an *n* × 1 column vector of external covariates for the *i*^th^ individual, *ϑ* is the vector of parameters associated with the baseline distribution, and *β*  is the vector of regression coefficients. When the parametric PH model is considered, the censored likelihood function can be expressed as

(49) $$\begin{array}{c} L\left(\vartheta ,\beta |D\right)=\overset{n}{\underset{i=1}{\prod }}{\left[f\left(t_{i}|\vartheta ,\beta ,x\right)\right]}^{\delta_{i}}{\left[s\left(t_{i}|\vartheta ,\beta ,x\right)\right]}^{1-\delta_{i}},\\ =\overset{n}{\underset{i=1}{\prod }}{\left[h\left(t_{i}|\vartheta ,\beta ,x\right).S\left(t_{i}|\vartheta ,\beta ,x\right)\right]}^{\delta_{i}}{\left[s\left(t_{i}|\vartheta ,\beta ,x\right)\right]}^{1-\delta_{i}},\\ =\overset{n}{\underset{i=1}{\prod }}{\left[h\left(t_{i}|\vartheta ,\beta ,x\right)\right]}^{\delta_{i}}\left[s\left(t_{i}||\vartheta |,|\beta |,|x\right)\right]\\ =\overset{n}{\underset{i=1}{\prod }}{\left[h\left(t_{i}|\vartheta ,\beta ,x\right)\right]}^{\delta_{i}}\text{exp}\left[-\int_{0}^{t}h\left(u\right)du\right]=\;\overset{n}{\underset{i=1}{\prod }}{\left[h\left(t_{i}|\vartheta \right)\exp\left(x{\;}^{\prime }\beta \right)\right]}^{\delta_{i}}\text{exp}\left[-\left[H\left(t_{i}|\vartheta \right)\exp\left(x{\;}^{\prime }\beta \right)\right]\right].\; \end{array}$$

An iterative optimization procedure (e.g., Newton–Raphson algorithm) can be used to obtain the maximum likelihood estimation $\hat{\vartheta }\text{ of}\vartheta$. Hypothesis testing and interval estimations of model parameters are possible due to the MLEs' approaching normality [7]. The natural logarithm of the likelihood function, so-called log-likelihood function can be written as follows:

(50) $$\begin{array}{c} \ell \left(\vartheta ,\beta |D\right)=\;\overset{n}{\underset{i=1}{\sum }}\delta_{i}\text{log}\left[h_{0}\left(t_{i}|\vartheta \right)+x_{i}^{\prime }\beta \right]-\overset{n}{\underset{i=1}{\sum }}H_{0}\left(t_{i}|\vartheta \right)\exp\left(x_{i}^{\prime }\beta \right),\; \end{array}$$

where *β* is a vector of the regression coefficients and *ϑ*′=(*k*, *α*, *η*) is the vector of the baseline distributional parameters.

In our case, if we assume that *a*=∑_*i*=1_^*n*^*δ*_*i*_, *p*_*i*_=exp(**x**_**i**_′*β*)  and *q*_*i*_=(*ηt*_*i*_)^*α*^. Use (36) for *h*_0_(.) and note that *H*_0_(*t*; *θ*)=∫_0_^*t*^*h*(*u*)*du* is the baseline cumulative hazard rate function as given by (37). The full log-likelihood function of the GLL PH model can be expressed as follows:

(51) $$\begin{array}{c} \ell \left(\vartheta |t\right)=a\text{log}\alpha +a\alpha \text{log}k+\left(\alpha -1\right)\overset{n}{\underset{i=1}{\sum }}\delta_{i}\text{log}t_{i}-\overset{n}{\underset{i=1}{\sum }}\delta_{i}\text{log}\left(1+q_{i}\right)+a\text{log}p_{i}-{\left(\frac{k}{\eta }\right)}^{\alpha }\overset{n}{\underset{i=1}{\sum }}p_{i}\log\left(1+q_{i}\right). \end{array}$$

To obtain the MLE's of ***θ*** ′=(*k*, *α*, *η*) and **β** ′, we can maximize (51) directly with respect to (*k*, *α*, *η*) and **β** ′ or we can solve the nonlinear equations below or the 1^st^ derivative of the log-likelihood function. The 1^st^ derivatives of the log-likelihood function are

(52) $$\begin{array}{c} \frac{\partial \ell \left(\tau |t\right)}{\partial \alpha }=\;\frac{a}{\alpha }+a\text{log}p_{i}+\overset{n}{\underset{i=1}{\sum }}\delta_{i}\text{log}t_{i}-\frac{1}{\alpha }\overset{n}{\underset{i=1}{\sum }}\delta_{i}q_{i}\left[\frac{\log\;q_{i}}{\left(1+q_{i}\right)}\right],\\ -\;{\left(\frac{k}{\eta }\right)}^{\alpha }\left(\frac{1}{\alpha }\right)\overset{n}{\underset{i=1}{\sum }}p_{i}q_{i}\left[\frac{\log\;q_{i}}{\left(1+q_{i}\right)}\right]-{\left(\frac{k}{\eta }\right)}^{\alpha }\text{log}\left(\frac{k}{\eta }\right)\overset{n}{\underset{i=1}{\sum }}p_{i}\log\left(1+q_{i}\right),\\ \frac{\partial \ell \left(\tau |t\right)}{\partial \eta }=\;-\left(\frac{\alpha }{\eta }\right)\overset{n}{\underset{i=1}{\sum }}\delta_{i}\left[\frac{q_{i}}{1+q_{i}}\right]-\left(\frac{\alpha }{\eta }\right){\left(\frac{k}{\eta }\right)}^{\alpha }\overset{n}{\underset{i=1}{\sum }}p_{i}\left[\frac{q_{i}}{1+q_{i}}\right]-\left(\frac{\alpha }{\eta }\right){\left(\frac{k}{\eta }\right)}^{\alpha }\overset{n}{\underset{i=1}{\sum }}p_{i}\log\left(1-\left[\frac{q_{i}}{1+q_{i}}\right]\right),\\ \frac{\partial \ell \left(\tau |t\right)}{\partial k}=\;\frac{a\alpha }{k}-\left(\frac{\alpha }{k}\right){\left(\frac{k}{\eta }\right)}^{\alpha }\overset{n}{\underset{i=1}{\sum }}p_{i}\log\left(1+q_{i}\right),\\ \frac{\partial \ell \left(\tau |t\right)}{\partial \beta_{j}}=\;\overset{n}{\underset{i=1}{\sum }}\delta_{i}Z_{ij}-{\left(\frac{k}{\eta }\right)}^{\alpha }\overset{n}{\underset{i=1}{\sum }}p_{i}\log\left(1+q_{i}\right)Z_{ij}\text{ for }j=1,2,\ldots ,p. \end{array}$$

To maximize log-likelihood functions, many software packages are available including proven optimization algorithms.

### 6.2. Bayesian Inference

In this section, Bayesian inference was used to estimate distributional parameters and regression coefficients using objective (or noninformative) priors to obtain proper posterior distributions.

#### 6.2.1. Priors for the Model Parameters

The specification of a prior distribution is a crucial aspect of any Bayesian inference. In parametric survival regression models, this is especially true. As a result, the prior scenario is built in this study using a noninformative independent prior for the parameters. The marginal prior distribution for every regression coefficient *β*_*m*, _*m*=1,…, 5,   is prompted as a normal distribution centred at zero and with a small precision, *N*(0,  0.001); on the other hand, a gamma distribution, gamma(10,10),   is chosen as the marginal prior distribution for the parameters of the GLL PH model due to the versatility of gamma distribution that include the noninformative priors (uniform) on the shape parameters. Many research publications in the literature, such as Danish and Aslam [23, 24], considered the assumption of the gamma priors for the baseline hazard parameters of PH models. Alvares et al. [1] took the assumption of independent gamma priors for the baseline hazard parameters of eight different parametric survival models. Muse et al. [22] used the assumption of independent gamma priors for the baseline hazard parameters of the of the generalized log-logistic AFT model, and other researchers take these priors into account.

For the baseline parameters of the GLL-PH model, we assume independent gamma priors.

(53) $$\begin{array}{c} p\left(\alpha \right)∼G\left(a_{1},b_{1}\right)=\;\frac{b_{1}^{a_{1}}}{\Gamma \left(a_{1}\right)}\alpha^{a_{1}-1}e^{-b_{1}\alpha };\;a_{1},b_{1},\alpha >0\;,\\ p\left(\eta \right)∼G\left(a_{2},b_{2}\right)=\;\frac{b_{2}^{a_{2}}}{\Gamma \left(a_{2}\right)}\eta^{a_{2}-1}e^{-b_{2}\eta };\;a_{2},b_{2},\eta >0\;,\\ p\left(k\right)∼G\left(a_{3},b_{3}\right)=\;\frac{b_{3}^{a_{3}}}{\Gamma \left(a_{3}\right)}k^{a_{3}-1}e^{-b_{3}k};\;a_{3},b_{3},k>0. \end{array}$$

Prior to that, we had the regression coefficients (assuming a normal distribution).

(54) $$\begin{array}{c} p\left(\beta {\;}^{\prime }\right)∼N\left(a_{4},b_{4}\right). \end{array}$$

The density function of the combined prior distribution of all unknown parameters and the regression coefficients are given as

(55) $$\begin{array}{c} p\left(\alpha ,k,\eta ,\;\beta {\;}^{\prime }\right)=\;p\left(\alpha \right)p\left(\eta \right)p\left(k\right)p\left(\beta {\;}^{\prime }\right). \end{array}$$

#### 6.2.2. The Likelihood Function

Unfortunately, the likelihood function of this generalized model is not implemented in BUGS and JAGS syntax. To generate the likelihood function, we use the “zero's trick” method that become popular in survival analysis and relies on Poisson modelling of expanded or reconstructed data [1]. The zero's trick approach works on the assumption that perhaps the contribution of a Poisson (*λ*) observable of zero is exp(−*λ*); if we set *λ*=−log(*f*(*t*_*i*_*|ϑ*, *β*, **x**)) with observable data as a vector of 0′*s*, we receive the right contributions of the proposed model [18].

#### 6.2.3. The Posterior Distribution

The joint posterior density function is equal to the multiplication of the prior distribution *p*(*α*, *k*, *η*,  **β** ′) and the likelihood function the joint posterior density function of the parameters *α*, *k*, *η*,  *an*  *d* *β*^**'**^ of GLL PH model given the data can be expressed using Bayes' theorem as

(56) $$\begin{array}{c} p\;\left(\alpha ,k,\eta ,\;\beta {\;}^{\prime }|x\right)\propto p\left(\alpha ,k,\eta ,\;\beta {\;}^{\prime }\right)L\left(\alpha ,k,\eta ,\;\beta {\;}^{\prime }\right),\\ p\;\left(\alpha ,k,\eta ,\;\beta {\;}^{\prime }|x\right)\propto \;p\left(\alpha \right)p\left(\eta \right)p\left(k\right)p\left(\beta {\;}^{\prime }\right)\;L\left(\alpha ,k,\eta ,\;\beta {\;}^{\prime }\right), \end{array}$$

where the first four terms on the equation represent the prior specification for the unknown parameters and are assumed to be independent and *L*(*α*, *k*, *η*,  *β*^**'**^) is the likelihood function expressed as follows:

(57) $$\begin{array}{c} L\left(\alpha ,k,\eta ,\;\beta {\;}^{\prime }\right)=\;\overset{n}{\underset{i=1}{\prod }}{\left[\frac{\alpha k{\left(kx\right)}^{\alpha -1}}{\left[1+{\left(\eta t\right)}^{\alpha }\right]}\;\exp\left(x{\;}^{\prime }\beta \right)\;\right]}^{\delta_{i}}\left[\exp\left(x{\;}^{\prime }\beta \right)\frac{k^{\alpha }}{\lambda^{\alpha }}\text{ log }\left[1+{\left(\lambda x\right)}^{\alpha }\right]\right],\;\\ p\;\left(\alpha ,k,\eta ,\;\beta {\;}^{\prime }|x\right)\propto \left\{\overset{p}{\underset{j=0}{\prod }}\pi \left(\beta_{j}\right)\right\}\alpha^{a_{1}+n-1}\eta^{a_{2}+n-1}k^{a_{3}+n-1}e^{-\left(b_{1}\alpha +b_{2}\eta +b_{3}k\right)}L\left(\alpha ,k,\eta ,\;\beta {\;}^{\prime }\right). \end{array}$$

The marginal distributions of the model parameters and the normalising joint posterior density function are difficult to calculate analytically, requiring high-dimensional integration and no close form inferences. To obtain estimates, we use McMC simulation methods, which involve sampling from the posterior distribution through using the Metropolis–Hastings Algorithm.

## 7. Simulation Study

In this section, we undertake an extensive simulation investigation to demonstrate the proposed parametric proportional hazard model's good Bayesian features. The parameter values are chosen to construct situations that mimic cancer population studies using a cancer that is severe (with a lower five-year survival rate), such as lung cancer [9, 25]. We demonstrate parameter estimation, the effect of censoring proportions, and sample sizes on inference in more detail.

### 7.1. Generating Survival Data from the PH Model

To simulate survival data for the GLL PH model, we use the inversion technique [40, 41] to generate survival data. This strategy is based on the link between a survival random variable's cumulative hazard rate function and a standard uniform random variable. When the cumulative hazard rate function has a closed form expression, it may be immediately applied, inverted, and readily implemented with R [26]. The censoring rates were estimated using administrative censorship at (1) Tc = 5 years, which resulted in around 20% censoring in all sets, and (2) Tc = 3 years, which resulted in about 30% censoring in all sets.

For the purposes of this simulation, we assume that survival times are distributed using the generalized log-logistic distribution (*α*, *η*, *k*). Using the reverse chf given in equation (41), lifetime data can be simulated as follows:

(58) $$\begin{array}{c} T\;=\;H{\;}_{0}^{-1}\left\{\frac{{\left(e^{{\left(\eta /k\right)}^{\alpha }\left[-\log\left(1-U\right)/e^{\beta x_{i}}\right]}\;-\;1\right)}^{1/\alpha }}{\eta }\right\},\; \end{array}$$

where *a*, *η*, and*k* > 0.

### 7.2. Simulation Design

The simulation analysis was carried out by conducting a series of simulations with different sample sizes (*n* = 100, and 300) sets and censoring proportions (Tc = 20 and 30 percentages), all based on the PH model in equation (1). The GLL PH model's true parameter vector is set as follows: (1) set I: distributional parameter values (*α*=1.5, *k*=0.75, and *η*=1.25) and covariates *β*=(0.75, −0.75, 0.5), (2) set II: distributional parameter values (*α*=1.5, *k*=0.95, and *η*=1.5) and covariates *β*=(0.75, −0.75,  0.5).

The values of the covariates were simulated as follows: (1) combination of uniform distributions with 0.25 probability on (30, 65), 0.35 probability on (65, 75), and 0.40 probability on (75, 85) years old was used to simulate the continuous covariate “age,” and (2) the binary covariates “treatment” and “gender” were both simulated using a 0.5 binomial distribution. We recommend that the reader can refer [9] for further details.

### 7.3. Posterior Analysis of the Simulated Data

We fitted the proposed PH model with GLL baseline hazard to assess its Bayesian properties in the simulation sets. With all censoring rates and different sample sizes, each simulation set was used to estimate the proposed PH model. JAGS software [27] was used to approximate posterior distributions using three parallel chains with 40,000 iterations each plus another 3,000 for the burn-in period. To minimize autocorrelation in the sequences, the chains were thinned further by storing every 10th draw.

### 7.4. Measures of Performance

The actual mean, standard deviation (SD), Naive standard error, bias, percentage of bias, coverage probability (CP), potential scale reduction factor $\left(\hat{R}\right),$ and the effective number of separate simulation draws were used to test the posterior distribution stability for the suggested PH model.

#### 7.4.1. Evaluating the Performance of the Estimators

We calculate the bias of the estimators using:

(59) $$\begin{array}{c} \text{Bias }\left(\hat{\theta }\right)=\frac{1}{N}\overset{N}{\underset{i=1}{\sum }}\left(\hat{\theta }-\theta \right). \end{array}$$

An underestimation is indicated by a negative bias, whereas an overestimation is shown by a positive bias.

#### 7.4.2. Accuracy of the Estimators

The mean square error (MSE) is a good indicator of overall accuracy and is calculated as follows:

(60) $$\begin{array}{c} \text{MSE }\left(\hat{\theta }\right)=\frac{1}{N}\overset{N}{\underset{i=1}{\sum }}{\left(\hat{\theta }-\theta \right)}^{2}. \end{array}$$

This metric determines how accurate the estimates are as follows. The lower the MSE, the more accurate the estimations of impacts.

The Naive standard error, which is calculated by dividing the posterior standard deviation by the square root of the sample size, is another accuracy metric. As a result, the smaller the standard error, the larger the sample size. The Naïve SE incorporates simulation error rather than posterior uncertainty.

(61) $$\begin{array}{c} \text{Naive SE}=\;\frac{\text{posterior SD}}{\sqrt{n}}. \end{array}$$

#### 7.4.3. Coverage

The 95 percent coverage probability (CP) is the percentage of *N* simulated data sets in which the true estimates were included in the 95 percent confidence interval. The more precise the estimations are, the closer the outcome is to a 95 percent coverage probability. The following is how CP is expressed:

(62) $$\begin{array}{c} CP=\hat{\theta }\mp 1.96\times SE\left(\hat{\theta }\right). \end{array}$$

#### 7.4.4. Convergence Diagnostics

Quantitatively, Gelman et al. [28] recommended that the acceptable limit of multivariate potential scale reduction factor (MPSRF) and potential scale reduction factor (PSRF) be near 1 $\hat{R}<1.1$, and the effective number of sample size simulation draws be greater than or equal to 100 for checking the convergence of McMC simulations. It is clear from the summary characteristics (Tables 1–4) that the PSRF is less than 1.1, that number of sample size simulation draws is larger than 100, and that Naive SE is smaller than the standard deviations (SD) for all of the distributional parameters and regression coefficients, as expected, indicating that the McMC algorithm has converged to the posterior distribution. Trace plots, autocorrelation plots, and Gelman plot diagnostics are the most common ways to judge the convergence of a McMC simulation graphically [28]. The McMC simulation has been achieved as evidenced by the trace plot, density plot, autocorrelation plot, and Gelman diagnostic plots for each distributional parameter and regression coefficients. That is, the McMC simulation for the GLL PH model explores the target posterior distribution appropriately.

### 7.5. Simulation Results

Tables 1–4 shows the simulation results for the posterior mean, bias, Naive standard error (SE), mean square error (MSE), coverage probability (CP), Gelman–Rubin diagnostic ($\left.\hat{R}\right)$, and the number of sample size simulation draws (no. of Eff) of the proposed PH model, and Figures 2–5 shows the visual summary for the convergence diagnostics.

Based on these findings, we may deduce that, as the sample size grows, the biases and MSE of the estimators decrease; also, the censoring proportion impacts the bias and MSE of the estimators, with larger censoring rates increasing the bias and MSE. The Gelman–Rubin diagnostic, on the other hand, as well as the number of efficiency sample size draws show that convergence has been attained. However, the estimators' coverage probability was close to 95%.

## 8. Practical Illustrations

In this section, two real-life survival data sets dealing with right-censored cancer data sets were considered to demonstrate the flexibility and applicability of the proposed GLL PH in modelling different survival data sets with different hazard rate shapes.

### 8.1. Data Set I: Lung Cancer Survival Data

#### 8.1.1. Data Description

In this section, we reanalyse the data set reported in [29] which is available in the R package survival. The Veterans Administration Lung Cancer Study Group followed up on *n* = 137 patients in this data set. For this clinical investigation, the censorship rate is around 6.5 percent (9 observations out of 137 were censored). The response and exploratory factors in this clinical trial are the time until death (in days), the number of months from diagnosis to study enrolment (diagt), age (in years), a history of previous lung cancer therapy (prior), and the trt = (treatment = conventional chemotherapy).

#### 8.1.2. Hazard Rate Shape

The hazard rate function appears to be unimodal or decreasing in Figure 6 based on the TTT plot (careful inspection reveals a slight indication of unimodality). The data could be evaluated with a model like the log-logistic distribution, which can accommodate decreasing or unimodal hazard rate forms. However, because the classical LL distribution is not closed under the PH framework, we employ the GLL distribution, which is closed and can encompass various hazard rate shapes. The box plot, histogram, and TTT plots are shown in Figure 6.

#### 8.1.3. Proportionality Assumption

There are two widely used methods for assessing the PH assumption: (1) graphical diagnostics based on (a) time-dependent variables [7] and (b) standardized Schoenfeld residuals [30] and (2) statistical tests. The standardized Schoenfeld residuals are used in this section to evaluate the PH assumption of the Cox model for each covariate included in the model. Based on Figure 7 and the significance threshold of 5%, there is no evidence to reject the proportional hazards assumption. As a result, we anticipate that the GLL PH model will provide a good fit when compared to the other existing parametric PH model employed in this study.

#### 8.1.4. Posterior Analysis

In this paper, we assume the noninformative independent framework with a normal prior *N*(0,  0.001) for *β*′*s* (regression coefficients) and an independent gamma prior for the distributional parameters *α* ~ *G*(*a*_1_, *b*_1_),  *η* ~ *G*(*a*_2_, *b*_2_),  and *k* ~ *G*(*a*_3_, *b*_3_) with hyperparameter values (*a*_1_=*b*_1_=*a*_2_=*b*_2_=*a*_3_=*b*_3_=10).

*(1) Numerical Summary*. We looked at various quantities of interest and their numerical values using the McMC sample of posterior properties for the generalized log-logistic proportional hazard model using the lung cancer data in this section.

The posterior summaries for the generalized log-logistic PH model parameters using Veterans lung cancer data sets are illustrated in Table 5. The probability that the corresponding parameter is +ve is given in the last row of Table 5. A posterior probability of 0.5 indicates that a positive parameter value is as likely as a negative one. Once we've saved the posterior sample for each model parameter, we can compute the posterior probability, for example, for *β*_1_, using mean  (*β*_1_ > 0).

*(2) Visual Summary*. We looked at density strip plots, trace plots, Gelman–Rubin diagnostic plots, Ergodic mean plots, and autocorrelation diagnostic plots in this section to get a visual description of the posterior properties. These plots and graphs provide a nearly comprehensive representation of the parameters' posterior uncertainty for the application of the lung cancer data sets.

*(3) Density Plots*. Density can be compared to the fundamental shapes associated with typical analytic distributions, and density plots can reveal behaviour in the tails, skewness, existence of multimodal behaviour, and data outliers.  Figure 8 illustrates the density plots for the GLL PH model parameters.

*(4) Time-Series Plots*. One of the most common diagnostics of an McMC simulation is a time series plot (or trace plot) [28].  Figure 9 shows that the McMC sampling process converges to the joint posterior distribution with no periodicity. As a result, we can say that the chains have converged.

*(5) Brooks–Gelman–Rubin (BGR) Convergence Diagnostic*. Gelman and Rubin [31] propose a convergence diagnostic technique to check the McMC algorithms simulation and is based on within chain variance and between chain variance. Gelman et al. [28] suggested that the limit of acceptance of potential scale reduction factor (PSRF) to be less than 1.1.  Figure 10 shows us that both PSRF and MPSRF are less than 1.1.

*(6) Running Mean Plots*. The running mean (also referred to Ergodic mean) is a well-known convergence diagnostic for McMC algorithms. The Ergodic mean is defined as the mean of all simulated sample values of up to a specific iteration [32]. Ergodic mean is used to observe the convergence pattern of the McMC chains.  Figure 11 shows us the Ergodic mean plots for the regression coefficients and the baseline hazard parameters. It is quite clear from the running mean time-series plots that the chains converge after *N* iterations to their mean values. However, these plots display only at the mean of the baseline hazard parameters and the regression coefficients and therefore are inadequate.

*(7) Autocorrelation Plots*. Although the autocorrelation plot is not strictly a convergence diagnostic tool, it does aid in indirectly assessing the convergence of the McMC simulation process [33].  Figure 12 shows the autocorrelation plots for all parameters and regression coefficients.

#### 8.1.5. Convergence of McMC Algorithm for the Veterans Lung Cancer Data Set

Computational developments in the previous few decades have recently emerged as a very useful instrument for employing McMC approaches [34] and fitting Bayesian survival regression models in time-to-event analysis. The complicated posterior distribution is sampled using the McMC algorithm. As a result, when an algorithm converges to the target posterior distribution, the Markov chain is stationary, and adding more samples will not change the shape and position of the posterior distribution's density in a meaningful way and hence will not change the estimations or other relevant outcomes.

*(1) Common Statistical Tests for Convergence Diagnostics*. The convergence of the McMC algorithm was checked quantitatively using conventional statistical tests for convergence diagnostics: (1) Brooks–Gelman–Rubin diagnostics [28]; (2) Raftery and Lewi diagnostics [35]; (3) Heidelberger and Welch's diagnostic tests [36]; and (4) Geweke diagnostics [37]. For more information about these tests, we can refer to [34].  Table 6 indicates the Geweke, Raftery–Lewis, and Heidelberger–Welch diagnostics for the GLL PH model parameters.

*(2) Graphical Techniques for Convergence Diagnostics*. Convergence diagnostics of an McMC algorithm can be examined graphically, including: (1) time series plot; (2) autocorrelation plot; (3) running mean plot; and (4) Gelman–Rubin plots. See Figures 9–12.

### 8.2. Data Set II: Larynx Cancer Data Sets

#### 8.2.1. Data Description

Lifetimes for 90 patients with larynx-cancer, according to the stage of cancer tumour (stages I–IV) are given in Table 7. The study time or time to death are recorded in months (where,  ^*∗*^ shows us the censored time). Alvares et al. [1]; Wang et al. [8]; and Christensen et al. [19] discussed the data from different aspects under different hazard-based regression models, and the data were first reported by [38]. The survival times (in months) of patients is illustrated in Table 7.

The other covariates of the data are as follows: (1) age (in years) at diagnosis and (2) the year of diagnosis. One goal of this study was to see if the age, year of diagnosis, and stage of cancer were associated with the death of patients with laryngeal cancer.

#### 8.2.2. Hazard Rate Shape

Based on the TTT plot, the hazard rate function is an increasing hazard in Figure 13. The data could be analyzed using a model such as the Weibull distribution, which can handle monotone hazard rate forms. We adopt the GLL distribution, which would be represented by the PH framework and can accommodate a variety of hazard rate shapes to see its applicability of the monotone (increasing) hazard rates. Figure 13 shows the box plot, histogram, and TTT plots.

#### 8.2.3. Proportionality Assumption

We investigated if the proportional hazards model could be used with this data set. The underlying assumption of the Cox model for each explanatory variable utilized in the model is depicted in Figure 14. With a significance level of 5%, there is no evidence to reject the PH assumption. As a result, we anticipate that the parametric PH model will provide a strong fit.

#### 8.2.4. Posterior Analysis

In this paper, we assume the noninformative independent framework with *N*(0,  0.001) for *β*′*s* (regression coefficients) and an independent gamma prior for the distributional parameters *α* ~ *G*(*a*_1_, *b*_1_),  *η* ~ *G*(*a*_2_, *b*_2_),  and *k* ~ *G*(*a*_3_, *b*_3_) with hyperparameter values (*a*_1_=*b*_1_=*a*_2_=*b*_2_=*a*_3_=*b*_3_=10).

*(1) Numerical Summary*. We looked at various quantities of importance as well as their numerical values using the McMC sample of posterior properties for the generalized log-logistic proportional hazard model considering the larynx data in this section.

The posterior summaries for the GLL-PH model parameters using larynx cancer data are illustrated in Table 8. The probability that the corresponding parameter is +ve is given in the last row of Table 8.

*(2) Visual Summary*. We looked at density strip plots (Figure 15), trace plots (Figure 16), Ergodic mean plots (Figure 17), autocorrelation plots (Figure 18), and Gelman–Rubin diagnostic plots (Figure 19), in this section, to get a visual description of the posterior properties. These plots and graphs provide a nearly comprehensive representation of the parameters' posterior uncertainty.

#### 8.2.5. Convergence Diagnostic Tests for the Larynx Cancer Data Using GLL PH Model

*(1) Statistical Tests*.  Table 9 indicates the Geweke, Raftery–Lewis, and Heidelberger–Welch diagnostics for the GLL PH model parameters.

*(2) Graphical Techniques*. Convergence diagnostics of an McMC algorithm for the larynx cancer data set are presented in Figures 16–19.

#### 8.2.6. Hazard Ratio (HR)

One of the most intriguing aspects of PH models is that the regression coefficients can be interpreted using the hazard ratio, which is preferred by many clinicians.

A key feature for PH models is the hazard ratio (HR), also known as the relative risk, between two individuals with covariate vectors **x**_1_ and **x**_2_. The HR is defined as

(63) $$\begin{array}{c} HR\left(x_{1},x_{2},h_{0},\beta \right)=\frac{h\left(t|x_{1}\;,h_{0},\beta \right)}{h\left(t|x_{2},h_{0},\beta \right)}=\;\exp\left[{\left(x_{1}-x_{2}\right)}^{T}\beta \right], \end{array}$$

which does not depend on time *t*. the hazard function in the numerator is equal to this constant HR times the hazard in the denominator, i.e.,

(64) $$\begin{array}{c} h\left(t|x_{1}\;,h_{0},\beta \right)=HR\;x\;h\left(t|x_{2},h_{0},\beta \right). \end{array}$$

Hence, the name “proportional hazards model” [19]. For example, the posterior distributions of the HR between two individuals of the same age and diagyr (year of diagnosis) but in different stages can be easily summarized.

Table 10 depicts the posterior characteristics of the hazard ratio between two men of the same age and diagnosis year (diagyr) but in different stages.

## 9. Bayesian Model Selection

In this study, we will use the deviance information criterion (DIC) to distinguish between the proposed models. DIC is a popular Bayesian model selection criterion. This criterion is available in most McMC packages [39]. The DIC is computed as follows:

(65) $$\begin{array}{c} \text{DIC}=\bar{D}+pD=\hat{D}+2pD, \end{array}$$

where $\bar{D}$ denotes the deviance's posterior mean and is a goodness of fit test for parametric survival models and *pD* calculates as the difference between $pD=\bar{D}-\hat{D}$, and it is denoted the effective number of proposed model parameters.

### 9.1. Data Set I

Table 11 displays some posterior characteristics for the three PH models (generalized log-logistic, Gompertz, and Weibull). Even though the estimates of the regression coefficient are significant compared, the flexibility provided by the GLL distribution's additional shape parameter contributes to its ultimate superiority over the Gompertz and Weibull models and the DIC shows us its goodness-of-fit and versatility comparing to the competing parametric PH models.

### 9.2. Data Set II

Table 12 displays some posterior characteristics for the three PH models (generalized log-logistic, Gompertz, and Weibull). Even though the estimates of the regression coefficient are significant compared, the flexibility provided by the GLL distribution's additional shape parameter contributes to its ultimate superiority over the Gompertz and Weibull models and the DIC demonstrates us its goodness-of-fit and versatility comparing to the competing parametric PH models.

## 10. Conclusion and Future Work

In this paper, we explored how to derive Bayesian estimates of the baseline hazard parameters and the regression coefficients of the parametric proportional hazard model with generalized log-logistic baseline hazard using right-censored survival data utilizing McMC approaches. The McMC techniques offer an alternative technique for estimating the parameters of the proposed model that is more flexible than frequentist techniques such as maximum likelihood estimation. Bayesian inference was performed with a variety of priors, and the convergence pattern was investigated using various diagnostic procedures.

To test the performance of the proposed parametric PH model, a comprehensive McMC simulation study was conducted. According to the simulation results, the PH model produces better results, with fewer absolute biases and MSEs for most regression coefficients and baseline distributional parameters. The behavior of the PH model in a generic PH regression situation comprising numerous covariates was also examined using synthetic right-censored data sets. Our findings indicate that the PH model performs well when handling with multiple factors. The paper's final analysis focused on a real-world application involving two well-known right-censored survival data sets for lung cancer and laryngeal cancer patients. In conclusion, the findings of the proposed parametric PH model show that it performs better and is superior to the other competing PH model, as well as indicating significant distributional parameters and regression coefficients.

Furthermore, for both simulation and real-data analysis, the regression coefficients were assumed to have a normal prior, and the baseline distribution parameters were assumed to have an independent gamma prior to compute the quantities of importance derived from the proposed model's posterior distribution. It has been attempted to create a visual summary and other essential graphs to aid in the interpretation of results and decision making. Finally, we hope that this paper will be an extension of the work of Khan and Khosa [11] and will encourage researchers who employ parametric hazard-based regression models to conduct their analyses using the Bayesian approach from the BUGs codes with the help of the R software's RJAGS package.

In terms of future work, we intend to produce an R package to fit the most prevalent parametric hazard-based regression models, including the PH model. The method given in this study can also be applied to multiple event scenarios, such as the competing risk model, and to survival data with a cure fraction rate. It can also be applied to joint model frameworks. Other types of censored and truncated observations, such as left censoring, interval censoring, and double censoring, could be used in future research. This is outside the scope of this study and will be addressed in future ones.

## Figures and Tables

**Figure 1:** Visual representation for the different hazard rate shapes of the GLL distribution with different values of the parameters.

**Figure 2:** Gelman diagnostics from a GLL PH framework with distributional parameters (*α*=1.5, *k*=0.75, and *η*=1.25), covariates *β*=(0.75, −0.75, 0.5), and *n*=300 and censoring proportion for 20 percentage.

**Figure 3:** Trace plots from a GLL PH framework with distributional parameters (*α*=1.5, *k*=0.75, and *η*=1.25), covariates *β*=(0.75, −0.75, 0.5), and *n*=300 and censoring proportion for 20 percentage.

**Figure 4:** Kernel density plots from a GLL PH framework with distributional parameters (*α*=1.5, *k*=0.75, and *η*=1.25) and covariates *β*=(0.75, −0.75, 0.5), and  *n*=300 and censoring proportion for 20 percentage.

**Figure 5:** Autocorrelation plots from a GLL PH framework with distributional parameters (*α*=1.5, *k*=0.75, and *η*=1.25), covariates *β*=(0.75, −0.75, 0.5), and *n*=300 and censoring proportion for 20 percentage.

**Figure 6:** TTT plot, box plot, and the histogram for the survival times of the lung cancer data sets.

**Figure 7:** The standardized Schoenfeld residuals from the data I—lung cancer data set, taking the test *p* value for each covariate into account.

**Figure 8:** Density plots for regression coefficients and distributional parameters from the Veterans lung cancer data set.

**Figure 9:** The time series plots for the baseline hazard parameters and the regression coefficients for the Veterans lung cancer data.

**Figure 10:** PSRF of the baseline hazard parameters and the regression coefficients for the Veterans lung cancer data.

**Figure 11:** The running mean plots for the baseline distributional parameters and regression coefficients for the Veterans lung cancer data set.

**Figure 12:** Autocorrelation plots for all the baseline distributional parameters and regression coefficients for the Veterans lung cancer data set.

**Figure 13:** TTT plot, box plot, and the histogram for the survival times of the larynx cancer data set.

**Figure 14:** The standardized Schoenfeld residuals from the data |—larynx cancer data set, taking the test *p* value for each covariate into account.

**Figure 15:** Density plots for the baseline hazard parameters and the regression coefficients for the larynx cancer data.

**Figure 16:** The time series plots for baseline hazard parameters and the regression coefficients for the larynx cancer.

**Figure 17:** The Ergodic mean plots for the baseline hazard parameters and regression coefficients for the larynx cancer data.

**Figure 18:** Autocorrelation plots for all the baseline hazard parameters and regression coefficients for the larynx cancer data.

**Figure 19:** PSRF of the baseline hazard parameters and the regression coefficients for the larynx cancer data.

**Table 1:** Simulation results from a GLL PH framework with distributional parameters (*α*=1.5, *k*=0.75, and *η*=1.25), covariates *β*=(0.75, −0.75, 0.5), and *n*=100.

Posterior properties							
True value $\left(\hat{\theta }\right)$	Posterior mean $\left(\hat{\theta }\right)$	Bias	Naïve SE	MSE	CP	$\hat{R}$	No. of eff
C = 20%							
*α*=1.50	1.506	0.006	0.001	0.032	0.032	1.000	3782
*β*_1_=0.75	0.837	0.087	0.002	0.057	0.935	1.001	3740
*β*_2_=−0.75	−0.695	0.055	0.001	0.011	0.945	1.000	3720
*β*_3_=0.50	0.480	0.020	0.002	0.049	0.920	1.002	3700
*η*=1.25	1.431	0.181	0.002	0.107	0.890	1.000	4039
*k*=0.75	0.720	0.030	0.001	0.013	0.935	1.001	4039

C = 30%							
*α*=1.50	1.463	−0.037	0.001	0.029	0.935	1.000	3802
*β*_1_=0.75	0.872	0.122	0.002	0.072	0.880	1.000	3823
*β*_2_=−0.75	−0.727	0.023	0.001	0.008	0.945	1.001	3761
*β*_3_=0.50	0.501	0.001	0.002	0.060	0.997	1.000	3700
*η*=1.25	1.575	0.325	0.002	0.193	0.851	1.002	3865
*k*=0.75	0.567	−0.183	0.001	0.045	0.911	1.000	4084

**Table 2:** Simulation results from a GLL PH framework with distributional parameters (*α*=1.5, *k*=0.75, and *η*=1.25), covariates *β*=(0.75, −0.75, 0.5), and  *n*=300.

Posterior properties							
True $\left(\hat{\theta }\right)$ Value	Posterior mean $\left(\hat{\theta }\right)$	Bias	Naïve SE	MSE	CP	$\hat{R}$	No. of eff
C = 20%							
*α*=1.50	1.449	−0.001	0.001	0.017	0.991	1.000	4017
*β*_1_=0.75	0.712	−0.038	0.001	0.019	0.946	1.000	3700
*β*_2_=−0.75	−0.723	0.027	0.000	0.003	0.956	1.000	3761
*β*_3_=0.50	0.483	−0.017	0.001	0.016	0.962	1.000	3782
*η*=1.25	1.309	0.059	0.002	0.070	0.923	1.001	4609
*k*=0.75	0.731	−0.019	0.001	0.012	0.941	1.001	4609

C = 30%							
*α*=1.50	1.527	0.027	0.001	0.021	0.945	1.000	4174
*β*_1_=0.75	0.726	−0.024	0.001	0.023	0.954	1.000	3660
*β*_2_=−0.75	−0.752	0.002	0.000	0.004	0.975	1.001	3802
*β*_3_=0.50	0.445	−0.055	0.001	0.023	0.937	1.001	3802
*η*=1.25	1.437	0.187	0.002	0.123	0.911	1.002	4434
*k*=0.75	0.847	0.097	0.001	0.023	0.907	1.003	4792

**Table 3:** Simulation results from a GLL PH framework with distributional parameters (*α*=1.75, *k*=0.95, and *η*=1.5), covariates *β*=(0.5, −0.85, 0.5), and *n*=100.

Posterior properties							
True $\left(\hat{\theta }\right)$ Value	Posterior mean $\left(\hat{\theta }\right)$	Bias	Naïve SE	MSE	CP	$\hat{R}$	No. of eff
C = 20%							
*α*=1.75	1.718	−0.032	0.002	0.038	0.942	1.000	3865
*β*_1_=0.50	0.523	0.023	0.002	0.051	0.955	1.000	3823
*β*_2_=−0.85	−0.817	−0.033	0.001	0.010	0.946	1.000	3720
*β*_3_=0.50	0.489	−0.011	0.002	0.050	0.981	1.000	3740
*η*=1.50	1.441	−0.059	0.002	0.068	0.931	1.000	4084
*k*=0.95	0.828	−0.122	0.001	0.147	0.925	1.001	4084

C = 30%							
*α*=1.75	1.717	−0.033	0.002	0.044	0.939	1.000	3802
*β*_1_=0.50	0.577	0.077	0.002	0.063	0.943	1.000	3823
*β*_2_=−0.85	−0.833	−0.017	0.001	0.009	0.971	1.000	3761
*β*_3_=0.50	0.474	−0.026	0.002	0.058	0.952	1.000	3700
*η*=1.50	1.625	0.125	0.002	0.143	0.919	1.002	3865
*k*=0.95	0.778	−0.172	0.001	0.213	0.908	1.001	4084

**Table 4:** Simulation results from a GLL PH framework with distributional parameters (*α*=1.75, *k*=0.95, and *η*=1.5), covariates *β*=(0.5, −0.85, 0.5), and *n*=300.

Posterior properties							
True $\left(\hat{\theta }\right)$ value	Posterior mean $\left(\hat{\theta }\right)$	Bias	Naïve SE	MSE	CP	$\hat{R}$	No. of eff
C = 20%							
*α*=1.75	1.756	0.006	0.001	0.023	0.978	1.000	3951
*β*_1_=0.50	0.503	0.003	0.001	0.040	0.991	1.000	3761
*β*_2_=−0.85	−0.827	−0.023	0.000	0.003	0.963	1.000	3761
*β*_3_=0.50	0.505	0.005	0.000	0.045	0.987	1.000	3740
*η*=1.50	1.519	0.019	0.002	0.107	0.942	1.000	4458
*k*=0.95	0.973	0.023	0.001	0.013	0.941	1.001	4458

C = 30%							
*α*=1.75	1.811	0.061	0.001	0.091	0.935	1.000	4011
*β*_1_=0.50	0.612	0.112	0.001	0.129	0.880	1.000	3978
*β*_2_=−0.85	−0.815	−0.035	0.000	0.004	0.945	1.000	4011
*β*_3_=0.50	0.521	0.021	0.001	0.063	0.997	1.000	3789
*η*=1.50	1.531	0.031	0.002	0.171	0.851	1.001	4458
*k*=0.95	0.990	0.040	0.002	0.145	0.911	1.002	4565

**Table 5:** Numerical summaries of posterior characteristics based on McMC sample of the GLL PH model for the lung cancer data set.

Characteristics	Pars						
	Alpha	*β*_1 _ (diagt)	*β*_2_ (age)	*β*_3_ (prior)	*β*_4_ (trt)	Eta	Kappa
Mean	1.317	0.002	−0.024	−0.015	−0.151	0.042	0.103
SD	0.173	0.010	0.008	0.021	0.178	0.015	0.049
Naïve SE	0.001	0.0001	0.0001	0.0002	0.001	0.0001	0.0004
Time series SE	0.003	0.0001	0.0001	0.0001	0.002	0.0002	0.001
Minimum	0.813	−0.046	−0.054	−0.109	−0.890	0.007	0.019
2.5^th^ percentile	1.023	−0.020	−0.040	−0.057	−0.500	0.019	0.040
Q1	1.194	−0.005	−0.029	−0.029	−0.271	0.031	0.068
Medium (Q2)	1.302	0.003	−0.024	−0.015	−0.150	0.040	0.092
Q3	1.422	0.010	−0.018	−0.0003	−0.029	0.051	0.125
97.5^th^ percentile	1.697	0.021	−0.007	0.027	0.193	0.078	0.231
Maximum	2.324	0.032	0.006	0.082	0.511	0.143	0.658
Mode	1.250	0.003	−0.028	−0.015	−0.150	0.035	0.075
Variance	0.030	0.0001	0.0001	0.001	0.032	0.0002	0.002
Skewness	0.550	−0.361	0.082	−0.058	−0.027	0.957	1.656
Kurtosis	0.558	0.152	0.011	0.001	−0.009	1.510	4.992
95% credible interval	(1.023, 1.697)	−0.020, 0.021)	(−0.040, −0.007)	(−0.057, 0.027)	(−0.500, 0.193)	(0.019, 0.078)	(0.040, 0.231)
P (.>0|data)	1.000	0.598	0.003	0.244	0.199	1.000	1.000

**Table 6:** Summaries for Raftery–Lewis's diagnostic, Geweke diagnostic, and Heidelberger–Welch diagnostics test of the GLL PH model parameters for the Veterans lung cancer data set.

Parameter	Geweke diagnostic	Diagnostics for the Raftery Lewis	Diagnostics for the Heidelberger–Welch		
	Pr > |z|	Dependency factor (I)	Stationarity test	*p* value	Halfwidth test
Alpha	−0.383	2.430	Passed	0.648	Passed
*β*_1_ (diagt)	0.820	1.030	Passed	0.337	Passed
*β*_2_ (age)	−0.272	3.640	Passed	0.613	Passed
*β*_3_ (prior)	−0.680	0.988	Passed	0.885	Passed
*β*_4_ (trt)	0.608	2.120	Passed	0.112	Passed
Eta	−1.436	1.160	Passed	0.178	Passed
Kappa	−0.142	3.500	Passed	0.506	Passed

**Table 7:** Survival times (in months) of patients with larynx cancer according to stages of tumour (1–4).

Stages	Survival time (^*∗*^ = indicating censoring)
Stage I (33 patients)	0.6, 1.3, 2.4, 2.5^*∗*^, 3.2, 3.3^*∗*^, 3.5, 3.5, 4.0, 4.0, 4.3, 4.5^*∗*^, 4.5^*∗*^, 5.3, 5.5^*∗*^, 5.9^*∗*^, 5.9^*∗*^, 6.0, 6.1^*∗*^, 6.2^*∗*^, 6.4, 6.5, 6.5^*∗*^, 6.7^*∗*^, 7.0^*∗*^, 7.4, 7.4^*∗*^, 8.1^*∗*^, 8.1^*∗*^, 9.6^*∗*^, 10.7^*∗*^
Stage II (17 patients)	0.2, 1.8, 2.0, 2.2^*∗*^, 2.6^*∗*^, 3.3^*∗*^, 3.6, 4.0^*∗*^, 4.3, 4.3^*∗*^, 5.0^*∗*^, 6.2, 7.0, 7.5^*∗*^, 7.6^*∗*^, 9.3^*∗*^
Stage III (patients)	0.3, 0.3, 0.5, 0.7, 0.8, 1.0, 1.3, 1.6, 1.8, 1.9, 1.9, 3.2, 3.5, 3.7^*∗*^, 4.5^*∗*^, 4.8^*∗*^, 4.8^*∗*^, 5.0, 5.0^*∗*^, 5.1^*∗*^, 6.3, 6.4, 6.5^*∗*^, 7.8, 8.0^*∗*^, 9.3^*∗*^, 10.1^*∗*^
Stage IV (13 patients)	0.1, 0.3, 0.4, 0.8, 0.8, 1.0, 1.5, 2.0, 2.3, 2.9^*∗*^, 3.6, 3.8, 4.3^*∗*^

**Table 8:** Numerical summaries of posterior characteristics based on McMC sample for GLL PH model for the larynx cancer data.

Characteristics	Pars							
	Alpha	*β*_1_ (stage 2)	*β*_2_ (stage 3)	*β*_3_ (stage 4)	*β*_4_ (age)	*β*_5_ (diagyr)	Eta	Kappa
Mean	1.539	−0.182	0.376	1.222	0.187	−0.111	0.869	0.336
SD	0.215	0.454	0.337	0.411	0.144	0.149	0.247	0.077
Naïve SE	0.002	0.004	0.003	0.004	0.001	0.001	0.002	0.001
Time series SE	0.002	0.004	0.003	0.004	0.001	0.001	0.003	0.001
Minimum	0.847	−1.975	−0.902	−0.531	−0.373	−0.730	0.197	0.112
2.5^th^ percentile	1.157	−1.108	−0.289	0.396	−0.091	−0.403	0.457	0.207
Q1	1.389	−0.480	0.152	0.952	0.089	−0.212	0.691	0.282
Medium (Q2)	1.524	−0.170	0.377	1.230	0.187	−0.112	0.846	0.328
Q3	1.668	0.128	0.605	1.498	0.284	−0.012	1.020	0.382
97.5^th^ percentile	2.005	0.667	1.030	2.010	0.476	0.181	1.412	0.507
Maximum	2.701	1.648	1.770	2.848	0.817	0.509	2.131	0.763
Mode	1.550	−0.100	0.300	1.300	0.150	−0.150	0.850	0.325
Variance	0.046	0.207	0.113	0.169	0.021	0.022	0.061	0.006
Skewness	0.447	−0.173	−0.041	−0.086	0.081	0.023	0.595	0.604
Kurtosis	0.511	0.068	0.010	0.070	0.102	0.027	0.514	0.656
95% credible interval	(1.157, 2.005)	(−1.108, 0.667)	(−0.289, 1.030)	(0.396, 2.010)	(−0.091, 0.476)	(−0.730, 0.181)	(0.197, 1.412)	(0.112, 0.507)
*P* (>0|data)	1.000	0.352	0.870	0.998	0.906	0.227	1.000	1.000

**Table 9:** Summaries for the Raftery–Lewis's, Geweke, and Heidelberger–Welch diagnostics test for the GLL PH model parameters for the right-censored larynx cancer data.

Parameter	Geweke diagnostic	Diagnostics for Raftery–Lewis	Diagnostics for the Heidelberger–Welch		
	Pr > |z|	Dependency factor (I)	*p* value	Stationarity test	Half width test
Alpha	1.083	1.020	0.787	Passed	Passed
*β*_1_ (stage 2)	−1.105	0.982	0.730	Passed	Passed
*β*_2_ (stage 3)	−0.333	1.060	0.497	Passed	Passed
*β*_3_ (stage 4)	0.969	1.030	0.053	Passed	Passed
*β*_4_ (age)	−0.800	1.020	0.680	Passed	Passed
*β*_5_ (diagyr)	−1.177	0.998	0.425	Passed	Passed
Eta	0.133	1.090	0.252	Passed	Passed
Kappa	0.317	1.150	0.189	Passed	Passed

**Table 10:** Posterior characteristics of the hazard ratio between two men of the same age and diagnosis year but in different tumour stages.

Posterior characteristics	Stages 3 and 4	Stages 2 and 4	Stages 2 and 3
Mean	0.467	0.280	0.638
Standard deviation (SD)	0.203	0.149	0.298
Naïve SE	0.001	0.001	0.002
Time series SE	0.002	0.001	0.002
2.5%	0.197	0.088	0.218
Lower quartile (Q1)	0.326	0.175	0.423
Medium (Q2)	0.425	0.250	0.585
Upper quartile (Q3)	0.564	0.349	0.791
97.5%	0.967	0.648	1.366

**Table 11:** Posterior properties summaries and the information criterion values for the considered GLL PH model and its competing models for the lung cancer data.

Summaries	Posterior characteristics				
Parametric competitive models	Parameter(s)	Posterior mean	Posterior SD	Pr (>|0|data)	HPD interval (95%)
GLL-PH model (DIC = 1505.165)					
	Alpha	1.317	0.173	1.000	(1.001, 1.661)
	*β*_1_ (diagt)	0.002	0.010	0.598	(−0.019, 0.021)
	*β*_2_ (age)	−0.024	0.008	0.003	(−0.039, −0.007)
	*β*_3_ (prior)	−0.015	0.021	0.244	(−0.057, 0.026)
	*β*_4_ (trt)	−0.151	0.178	0.199	(−0.505, 0.186)
	Eta	0.042	0.015	1.000	(0.016, 0.073)
	Kappa	0.103	0.049	1.000	(0.029, 0.200)

Weibull-PH model (DIC = 1521.310)					
	Alpha	0.744	0.048	1.000	(0.654, 0.842)
	*β*_1_ (diagt)	0.005	0.010	0.648	(−0.018, 0.024)
	*β*_2_ (age)	−0.025	0.007	0.001	(−0.039, −0.010)
	*β*_3_ (prior)	−1.027	0.021	0.102	(−0.068, 0.015)
	*β*_4_ (trt)	−0.252	0.180	0.080	(−0.593, 0.108)
	Kappa	0.206	0.090	1.000	(0.060, 0.388)

Gompertz-PH model (DIC = 1556.407)					
	Alpha	1.134	0.311	1.000	(0.567, 1.746)
	*β*_1_ (diagt)	0.021	0.009	0.984	(0.003, 0.039)
	*β*_2_ (age)	0.027	0.006	1.000	(0.014, 0.039)
	*β*_3_ (prior)	−0.056	0.023	0.006	(−0.099, −0.012)
	*β*_4_ (trt)	−0.136	0.182	0.228	(−0.494, −0.211)
	Kappa	0.001	0.0002	1.000	(0.001, 0.002)

**Table 12:** Posterior properties summaries and the information criterion values for the considered GLL PH model and its competing models for the larynx cancer data.

Summaries	Posterior characteristics				
Parametric competitive models	Parameter(s)	Posterior mean	Posterior SD	Pr (>|0|data)	HPD interval (95%)
GLL-PH model (DIC = 294.412)					
	Alpha	1.539	0.215	1.000	(1.157, 2.005)
	*β*_1_ (stage 2)	−0.182	0.454	0.352	(−1.108, 0.667)
	*β*_2_ (stage 3)	0.376	0.337	0.870	(−0.289, 1.030)
	*β*_3_ (stage 4)	1.222	0.411	0.998	(0.396, 2.010)
	*β*_4_ (age)	0.187	0.144	0.906	(−0.091, 0.476)
	*β*_5_ (diagyr)	−0.111	0.149	0.227	−0.730, 0.181)
	Eta	0.869	0.247	1.000	(0.197, 1.412)
	Kappa	0.336	0.077	1.000	(0.112, 0.507)

Weibull-PH model (DIC = 296.776)					
	Alpha	0.908	0.105	1.000	(0.713, 1.118)
	*β*_1_ (stage 2)	−0.380	0.446	0.198	(−1.275, 0.468)
	*β*_2_ (stage 3)	0.174	0.318	0.711	(−0.483, 0.781)
	*β*_3_ (stage 4)	1.095	0.393	0.997	(0.329, 1.857)
	*β*_4_ (age)	0.176	0.141	0.899	(−0.092, 0.461)
	*β*_5_ (diagyr)	−0.012	0.146	0.468	(−0.294, 0.274)
	Kappa	0.154	0.041	1.000	(0.081, 0.236)

Gompertz-PH model (WAIC = 297.560)					
	Alpha	0.134	0.031	1.000	(0.076, 0.196)
	*β*_1_ (stage 2)	−0.138	0.455	0.392	(−1.040, 0.737)
	*β*_2_ (stage 3)	0.393	0.328	0.886	(−0.252, 1.041)
	*β*_3_ (stage 4)	1.544	0.397	1.000	(0.776, 2.308)
	*β*_4_ (age)	0.206	0.149	0.919	(−0.084, −0.501)
	*β*_5_ (diagyr)	0.075	0.155	0.685	(−0.230, 0.374)
	Kappa	0.552	0.186	1.000	(0.227, 0.919)

## Data Availability

The data used to support the findings of this study are included within the article.
